The article "Interferon-β Induces Cellular Senescence in Cutaneous Human Papilloma Virus-Transformed Human Keratinocytes by Affecting p53 Transactivating Activity" was retracted in 2019. Reasons: manipulated images; duplicated images.

# Interferon-β Induces Cellular Senescence in Cutaneous Human Papilloma Virus-Transformed Human Keratinocytes by Affecting p53 Transactivating Activity

**DOI:** 10.1371/journal.pone.0036909

**Published:** 2012-05-16

**Authors:** Maria V. Chiantore, Serena Vannucchi, Rosita Accardi, Massimo Tommasino, Zulema A. Percario, Gabriele Vaccari, Elisabetta Affabris, Gianna Fiorucci, Giovanna Romeo

**Affiliations:** 1 Department of Infectious, Parasitic and Immune-mediated Diseases, Istituto Superiore di Sanità, Rome, Italy; 2 Infections and Cancer Biology Group, International Agency for Research on Cancer-WHO, Lyon, France; 3 Department of Biology, University of Rome 3, Rome, Italy; 4 Department of Veterinary Public Health and Food Safety, Istituto Superiore di Sanità, Rome, Italy; 5 Institute of Molecular Biology and Pathology, CNR, Rome, Italy; 6 Department of Medico-Surgical Sciences and Biotechnologies, Sapienza University, Rome, Italy; Consiglio Nazionale delle Ricerche (CNR), Italy

## Abstract

Interferon (IFN)-β inhibits cell proliferation and affects cell cycle in keratinocytes transformed by both mucosal high risk Human Papilloma Virus (HPV) and cutaneous HPV E6 and E7 proteins. In particular, upon longer IFN-β treatments, cutaneous HPV38 expressing cells undergo senescence. IFN-β appears to induce senescence by upregulating the expression of the tumor suppressor PML, a well known IFN-induced gene. Indeed, experiments in gene silencing via specific siRNAs have shown that PML is essential in the execution of the senescence programme and that both p53 and p21 pathways are involved. IFN-β treatment leads to a modulation of p53 phosphorylation and acetylation status and a reduction in the expression of the p53 dominant negative ΔNp73. These effects allow the recovery of p53 transactivating activity of target genes involved in the control of cell proliferation. Taken together, these studies suggest that signaling through the IFN pathway might play an important role in cellular senescence. This additional understanding of IFN antitumor action and mechanisms influencing tumor responsiveness or resistance appears useful in aiding further promising development of biomolecular strategies in the IFN therapy of cancer.

## Introduction

The group of cellular proteins known as Interferons (IFNs) appeared to be expressed in infected cells as an early response to viral infection but, in addition to their antiviral activity, IFNs also have a profound effect on cell growth [1].

IFN-α2 was the first human protein shown to be effective for cancer treatment and the first economically viable clinical product developed from recombinant DNA technology in cancer therapy.

The article "Interferon-β Induces Cellular Senescence in Cutaneous Human Papilloma Virus-Transformed Human Keratinocytes by Affecting p53 Transactivating Activity" was retracted in 2019. Reasons: manipulated images; duplicated images.

Antitumor activity of IFNs is probably exerted through direct and indirect mechanisms. It is conceivable that numerous direct effects play a central role in the overall antitumor response, such as down-regulation of oncogene expression, induction of differentiation, inhibition of cell cycle progression and induction of tumor suppressor genes, and programmed cell death [2]. However, additional understanding of IFN antitumor action and mechanisms influencing tumor responsiveness or resistance appears necessary to aid further promising development of biomolecular strategies in IFN therapy of cancer.

The most extensively studied anticancer treatment-induced mechanism is apoptotic programmed cell death. Nevertheless, the correlation between the induction of apoptosis and drug response cannot explain the overall tumor cell sensitivity [3]. Numerous recent studies have shown that in cells where apoptosis is blocked, non-apoptotic cell death or irreversible cell growth arrest, namely senescence, can be activated as potential tumor-suppressor mechanisms [4]. The concept of senescence is applied in general to the irreversible proliferative arrest of cells caused by various stresses [5] including oxidative damage, telomere dysfunction, and DNA damage. One particularly relevant source of stress in tumor cells is derived from the aberrant proliferative signals of oncogenes which may trigger senescence through a process known as oncogene-induced senescence, functioning as a potential tumor suppressor mechanism.

Senescent cells are identified *in vitro* by distinctive morphological changes, such as large cell size, flat vacuolated morphology, the inability to synthesize DNA, the formation of domains of heterochromatin called Senescence-Associated Heterochromatin *Foci* (SAHF) and the expression of a Senescence-Associated β-galactosidase activity (SA-β-gal) [6], [7]. One of the earliest steps in the senescence programme is the translocation of histone chaperone HIRA (Histone Repression factor A) into promyelocytic leukemia (PML) nuclear bodies (NBs), but the role played by HIRA localization into PML bodies has not yet been identified. PML bodies are nuclear structures known to serve as sites of protein modification and the assembly of macromolecular regulatory complexes, and have been extensively implicated in the induction of senescence and apoptosis [8], [9].

Consistent with its role in tumor suppression, the critical senescence pathways converge on the two major tumor suppressor genes p53 and pRb, whose mutations or inactivation are most common in all cancers [10].

Abrogation of senescence can be achieved by SV40 large T, a combination of HPV oncoproteins E6 and E7, E1A and MDM2 coexpression or small interfering RNA against pRb and p53 [11]. Tumors initiated by loss of p53 can be eliminated by senescence induced by p53 restoration, tumor regression being achieved through an innate immune response that leads to the clearance of senescent cells [12], [13]. Cellular senescence results in altered gene expression including IFNs and their related genes [14]. PML is known to be regulated by the interferon pathway via the STAT transcription factors [15]. IFN also regulates many other components of PML nuclear bodies, suggesting that in conjunction they mediate the antiviral and antiproliferative activities of this cytokine [9]. Cellular senescence is induced in human fibroblasts by prolonged IFN-β treatment through DNA damage signaling and a p53-dependent pathway [16]. IFN-α also induces replicative senescence in endothelial cells after continuous stimulation [17]. Taken together, these studies suggest that signaling through the IFN pathway might play an important role in cellular senescence.

The article "Interferon-β Induces Cellular Senescence in Cutaneous Human Papilloma Virus-Transformed Human Keratinocytes by Affecting p53 Transactivating Activity" was retracted in 2019. Reasons: manipulated images; duplicated images.

Human Papilloma Viruses (HPVs) are small DNA viruses involved in the development of both benign and malignant lesions localised in different anatomic districts, that are able to replicate exclusively in the stratified squamous cutaneous and mucosal epithelium. More than 100 different HPV types have been isolated so far, and they can be sub-grouped into cutaneous or mucosal according to their ability to infect the skin or the mucosa of the genital or upper-respiratory tracts [18]. To date, the causative association between mucosal high risk-HPV and cervical carcinoma has been clearly demonstrated. It is well known that the expression of E6 and E7 viral oncoproteins is a common feature of cervical cancer cells and is strongly implicated in the process of cancer development, E6 and E7 principally targeting and inhibiting p53 and pRb tumor suppressor proteins, respectively [19]. Emerging lines of evidence support the involvement of the cutaneous HPV types belonging to the beta genus in non melanoma skin cancer (NMSC). However, although the role of beta HPV types in NMSC in Epidermodysplasia verruciformis (EV) patients is well accepted, their involvement in skin carcinogenesis in the general population is not entirely proven. The transforming properties of the majority of cutaneous HPV types have been poorly investigated. Tommasino and co-workers [20] have shown that HPV38 E7 appears to act similarly to HPV16 E7, by binding to pRB and promoting its degradation via the proteasome pathway. On the contrary, HPV38 E6 oncoprotein differs from mucosal high risk HPV E6 proteins in the mechanism by which it counteracts p53 activity. The expression of HPV38 E6 and E7 in human keratinocytes induces the stabilization of p53, which in turn selectively activates transcription of ΔNp73, a p53 inhibitor [21]. High ΔNp73 levels have been found in a number of human malignancies including cancers of the breast, prostate, liver, lung and thyroid [22]. Recently, it has been shown that IFN-α reduces ΔNp73 levels in Huh7 hepatoma cells, and this effect correlates to increased susceptibility to IFN-α triggered apoptosis [23].

The article "Interferon-β Induces Cellular Senescence in Cutaneous Human Papilloma Virus-Transformed Human Keratinocytes by Affecting p53 Transactivating Activity" was retracted in 2019. Reasons: manipulated images; duplicated images.

Here, we show that prolonged treatment with IFN-β induces senescence in cutaneous HPV38-transformed keratinocytes. PML is essential in IFN-β induction of senescence in HPV38-transformed keratinocytes, and both p53 and p21 pathways contribute to the execution of the phenomenon. p53 colocalyzes with IFN-β-induced PML into PML Nuclear Bodies. By recruitment of p53 into NBs, IFN-β can modulate p53 post-translational modification at specific phosphorylation and acetylation sites and downregulate ΔNp73 expression, leading to the recovery of p53 transactivating activity of selected target genes involved in cell proliferation control.

## Results

### IFN-β Inhibits Cell Proliferation of K38 and K16 Cells

Keratinocytes expressing E6 and E7 proteins of HPV-38 and HPV-16, referred to as K38 and K16 respectively, were obtained as described [20].

To test whether IFN-β could affect proliferation of both transformed keratinocytes, K-38 and K-16 cells were treated with IFN-β for several time points and the amounts of viable cells were revealed. As shown in Fig. 1A, proliferation of both cell lines was strongly affected by IFN-β.

**Figure 1:** IFN-β affects cell proliferation in K16 and K38 cells. (A) IFN-β inhibits cell proliferation in K16 and K38 cells. Cells were seeded in triplicate at 10^5^ cells per 35 mm dish and, after 24 h, IFN-β was added to the cultures for the indicated times. IFN-β treated and control cells were counted in a hemocytometer and viability was evaluated by trypan blue exclusion. Data represent means ± s.d. of three independent experiments. ** = p<0.01; *** = p<0.001. **(**B**)** IFN-β treatment differently affects cell cycle progression of K16 and K38 cells. K16 and K38 cells were treated with IFN-β for the indicated time points. DNA staining was performed by incubating cells in PBS containing 0.18 mg/ml propidium iodide and 0.4 mg/ml DNase-free RNase. Cells were analysed on a FACScan flow cytometer. DNA profiles, derived from one representative experiment of three performed, are shown. (C) IFN-β treatment differently affects DNA synthesis in K16 and K38 cells. To determine the number of S-phase nuclei, cells were plated in triplicate at 10^5^ cells per 35 mm dish, treated with IFN-β for different time points and incubated with 50 µM BrdU for the last 5 hours. BrdU treated samples were then fixed and stained with an anti-BrdU monoclonal antibody followed by a rhodamine conjugated goat anti-mouse antibody. BrdU-positive cells were counted under a fluorescence microscope. Data represent means ± s.d. of three independent experiments.

The article "Interferon-β Induces Cellular Senescence in Cutaneous Human Papilloma Virus-Transformed Human Keratinocytes by Affecting p53 Transactivating Activity" was retracted in 2019. Reasons: manipulated images; duplicated images.

To exclude that the antiproliferative effect of IFN-β could be due to downregulation of E6/E7 expression, we checked HPV-38 and HPV-16 E6 and E7 mRNA levels by RT-PCR. No significant variations were observed in either E6 or E7 expression in K38 and K16 cells upon treatment with IFN-β for different time points (data not shown).

We previously demonstrated that IFN-β exerts its antiproliferative effect on high-risk HPV-positive cell lines by lengthening cell cycle S-phase progression [24]. We analyzed cell cycle distribution of K38 and K16 cells after treatment with IFN-β for several time points. Both cell lines showed a significant augment of S-phase cell amount starting from 48 h of treatment. Interestingly, in K16 cells S-phase cell accumulation increased with time whereas in K-38 cells the S-phase increase was followed by an augment of G1 population (Fig.1B).

K16 and K38 cells were pulse-labelled with BrdU for 5 h and analysed for BrdU incorporation. As with what was observed in SiHa and other mucosal high-risk HPV-positive cell lines [24], an increased number of BrdU-positive cells reflecting an S-phase cell accumulation was revealed in IFN-β treated K16 populations. On the contrary, in K-38 samples the number of cells incorporating BrdU upon IFN-β treatment appeared clearly reduced (Fig. 1C).

### IFN-β Induces Cellular Senescence in K38 but Not in K16 Cells

To study apoptosis and senescence induction, specific assays were performed. Annexin-V externalization assay showed no significant increase of apoptosis in either cell types after IFN-β treatment (data not shown). Senescent cells were quantified by counting cells displaying β-galactosidase activity at pH 6.0 (SA-βgal). This lysosomal hydrolase is elevated in senescent cells as a result of lysosomal activity at suboptimal pH, which is detectable only in senescent cells due to an increase in lysosomal content. Interestingly, increasingly high percentages of senescent cells were observed exclusively in K38 cells transformed by E6 and E7 proteins of cutaneous HPV genotype, starting from 4 days of IFN-β treatment, compared to control keratinocytes (LXSN), K16 cells and mucosal high risk HPV-positive cell lines (Fig. 2A, B, and C).

**Figure 2:** IFN-β induces senescence in K38 cells. (A) Control keratinocytes (LXSN), K16, K38 cells and high risk HPV-positive squamous carcinoma cell lines ME-180, Caski, HeLa and SiHa were treated with IFN-β for 4 days and senescent cells were quantified by counting cells displaying senescent-associated β-galactosidase (SA-βgal) activity at pH 6.0. (B) Percentage of senescent cells in K16 and K38 cells treated with IFN-β for different time points. (C) SA-βgal-positive K38 blue cells observed under a light microscope after 4 days of IFN-β treatment. * = p<0.05; *** = p<0.001.

The article "Interferon-β Induces Cellular Senescence in Cutaneous Human Papilloma Virus-Transformed Human Keratinocytes by Affecting p53 Transactivating Activity" was retracted in 2019. Reasons: manipulated images; duplicated images.

### Involvement of PML, p53 and p21 in Cell Senescence Induced by IFN-β in K-38 Cells

It is known that important senescence regulators are found in IFN-inducible genes. In addition, it has been reported that prolonged IFN-β stimulation can induce senescence in normal cells through the activation of a DNA damage response triggered by an ATM-chk2-p53 pathway [16]. We asked whether IFN-β could induce the senescence phenotype in K38 cells through the involvement of PML and the activation of p53, thus counteracting the inhibitory action exerted on p53 by HPV-38 E6/E7 expression. We analysed the protein levels of PML, p53 and p21, upon IFN-β treatment, and the respective involvement in senescence through RNA silencing (siRNA) technique. Three different siRNAs were used for PML, p53 and p21 genes. Upon IFN-β treatment, PML was up-regulated as well as p21 (Fig. 3). On the other hand in K16 cells, even if IFN-β treatment induces PML expression, it is not detectable any increase in p21 protein levels (data not shown).

**Figure 3:** IFN-β affects the expression of proteins involved in senescence in K38 cells. Western blot analysis of PML, p53 and p21 expression in K38 treated with IFN-β for different time points. Whole cell extracts were resolved on SDS-PAGE and transferred onto PVDF membrane. Immunoblotting was performed as reported in M&M.

PML seems to be an essential component of senescence response in K38 cells, since, when PML expression is inhibited by specific siRNAs (Fig. 4A), IFN-β-induced senescence is strongly reduced (Fig. 4D). p21 silencing (Fig. 4C) partially affects IFN-β-induced senescence (Fig. 4D), while p53 silencing (Fig. 4B) appears much more effective (Fig. 4D), suggesting that different p53 targets may be involved in IFN-β-induced senescence in K38 cells and different pathways may cooperate towards this phenomenon.

**Figure 4:** Effect of PML, p53 and p21 silencing on senescence induction by IFN-β in K38 cells. PML (A), p53 (B) and p21 (C) were silenced by specific small interfering RNAs and protein expression was analyzed by Western blot in cells treated with IFN-β for 4 days. (D) Senescence induction by IFN-β (4 days treatment) was evaluated by SA-βgal staining. * = p<0.05; ** = p<0.01.

The article "Interferon-β Induces Cellular Senescence in Cutaneous Human Papilloma Virus-Transformed Human Keratinocytes by Affecting p53 Transactivating Activity" was retracted in 2019. Reasons: manipulated images; duplicated images.

### PML Target Proteins Colocalyze in PML Nuclear Bodies

It is known that PML recruits into NBs p53 and different proteins involved in p53 post-translational modifications that are critical for the activation of p53 and for the selection of target genes [25]. We studied colocalization of PML with p53 and ΔNp73 through confocal microscopy analyses of K38 cells treated with IFN-β for different time points. Fig. 5 shows that p53 (A) and ΔNp73 (B) colocalyze with IFN-β-induced PML into PML NBs. On the other hand, colocalization is not detectable after PML silencing (data not shown).

**Figure 5:** p53 and ΔNp73 co-localyze with IFN-β-induced PML into PML Nuclear Bodies. (A,B) For confocal microscopy analysis, K38 cells were cultured on glass bottom dishes (MatTek Corporation) and treated with IFN-β for 4 days. Cells were then fixed in PBS 4% paraformaldehyde for 30 min on ice, immuno-fluorescence labelling was performed as described in Materials and Methods and sample were analyzed using confocal microscope (Leica TCS SP5).

### Post-translational Modification of p53 by IFN-β

The expression of HPV38 E6 and E7 in human keratinocytes induces the stabilization of p53, as shown by WB analysis of p53 in K38 cells compared with control keratinocytes (LXSN), K16 cells and high risk HPV-positive cell lines SiHA and ME-180 (Fig. 6A). This p53 stabilization can be related to increased phosphorylation [21] and acetylation (Fig. 6C).

**Figure 6:** IFN-β effect on p53 post-translational modification and expression of its target genes. (A) WB analysis of p53 in control keratinocytes (LXSN), K16 and K38 cells and in high risk HPV-positive squamous carcinoma cell lines SiHa and ME-180 treated with IFN-β for 48 h. (B) WB analysis of p53 phosphorylated at different phosphorylation sites. (C) WB analysis of acetylated p53. (D) WB analysis of phosphorylated and acetylated p53 and ΔNp73 in K38 cells silenced by PML siRNA and treated with IFN-β for 48 h. (E) WB analysis of ΔNp73 in K38 cells treated with IFN-β for different time points. Whole cell extracts were resolved on SDS-PAGE and transferred onto PVDF membrane. Immunoblotting was performed as reported in M&M. (F) Real time PCR analysis of Bax and Pig3 was carried out on K38 cells treated with IFN-β for 48 h, also in the presence of PML siRNA. NT  =  not transfected. * = p<0.05; ** = p<0.01.

In this respect, we may hypothesize that IFN-β, through PML up-regulation, can lead to the recovery of p53 transactivating activity of target genes involved in cell proliferation control. Therefore p53 phosphorylation and acetylation status was analyzed in K38 cells treated with IFN-β. IFN-β modulates p53 phosphorylation status at different phosphorylation sites (Ser-6, Ser-15, Ser-46, Ser-392, Fig. 6B **)** while acetylation is mainly downregulated in Lys-320 (Fig. 6C). Ser-6, Ser-392, and Lys-320 seem to be the most important p53 post-translational modifications involved in IFN-β-induced senescence in K38 cells. In fact, when PML expression is silenced, IFN-β is not able to modulate p53 Ser-6, Ser-392, and Lys-320 status (Fig. 6D).

The article "Interferon-β Induces Cellular Senescence in Cutaneous Human Papilloma Virus-Transformed Human Keratinocytes by Affecting p53 Transactivating Activity" was retracted in 2019. Reasons: manipulated images; duplicated images.

Accardi *et al*. [21] reported that p53 stabilization in K38 cells leads to transcriptional activation of ΔNp73, a p53 inhibitor, able to inhibit p53 transactivation of genes involved in cell growth suppression. It has been shown that IFN-α reduces ΔNp73 levels in Huh7 hepatoma cells and this effect correlates to increased susceptibility to IFN-α triggered apoptosis [23]. We observed that in K38 cells, IFN-β treatment downregulates ΔNp73 mRNA levels (data not shown). The ΔNp73 protein expression appears to be reduced upon IFN-β treatment (Fig. 6E), probably as a result of the p53 post-translational modifications induced by IFN-β. In fact, when PML expression is silenced, ΔNp73 protein levels are not downregulated by IFN-β (Fig. 6D).

Real time PCR array results indicate that some genes involved in senescence and growth control are IFN-β-upregulated (Fig.6F). In particular, the observed induction of p53 target genes Bax and Pig3 indicates that IFN-β treatment leads to the recovery of p53 transactivating activity of selected target genes involved in the control of cell proliferation. In fact, it has been reported that modification of specific p53 phosphorylation and acetylation sites may correlate to the transactivation of growth related genes, suggesting a tissue and promoter-specific p53 activity regulation [26]. PML depletion reduces IFN-β induction of Bax and Pig3 in K-38 cells (Fig.6F), indicating the role of PML in the ability of IFN-β to recover p53 transactivation activity of specific target genes.

## Discussion

IFNs were the first successful biological therapy for human malignancy and currently there are several approved IFN cancer therapies. Clinical effectiveness of different IFN subtypes in treatment of various forms of cancer has been extensively reviewed [1]. Better definition of therapeutic molecular targets appears to be critical to fully realize the potential of IFNs in oncology and further understand the mechanisms of antitumor action of the IFN family.

Senescence is a permanent cell cycle arrest that is resistant to growth factors and other signals that induce cell proliferation. It has been proposed that senescence prevents cancer in the early stages of its development [6]. Tumor suppressors such as p53, pRb and PML are critical regulators of senescent programme [10], [25], and genes required for senescence are often found to be mutated in human cancers. Cellular senescence is induced in human fibroblasts by prolonged IFN-β treatment through DNA damage signaling and a p53-dependent pathway [16]. IFN-α also induces replicative senescence in endothelial cells after continuous stimulation [17], and treatment with IFN-γ induces cellular senescence in young human umbilical vascular endothelial cells [27]. However, whether induction of senescence is sufficient to repress tumor *in vivo* is controversial. Recent reports showed that conditional restoration of p53 in mice with hepatocarcinomas, sarcoma or lymphoma is able to promote tumor regression [13], [12]. In addition, it has been reported that HeLa cells cease proliferation and undergo senescence by introduction of the bovine papillomavirus E2 gene that inhibits the expression of the HPV18 E7 gene [28]. Antisense sequences directed against HPV16 E6 and E7 genes transfected in SiHa cells contributed to apoptosis and senescence [29].

The article "Interferon-β Induces Cellular Senescence in Cutaneous Human Papilloma Virus-Transformed Human Keratinocytes by Affecting p53 Transactivating Activity" was retracted in 2019. Reasons: manipulated images; duplicated images.

In contrast to mucosal high-risk HPV types, the involvement of cutaneous HPV types in human carcinogenesis is still unclear. Cutaneous HPV types that belong to the beta genus of the HPV phylogenetic tree were first isolated in patients suffering from EV, a rare autosomal recessive cancer-prone genetic disorder, and are consistently detected in NMSC from EV, immunocompromised and normal individuals [30]. The transforming properties of the majority of the cutaneous HPV types have been poorly investigated. It has been reported that cutaneous HPV5 E6 protein targets and abrogates Bak function by promoting its proteolitic degradation both *in vitro* and in regenerated epithelium [31]; however, regulation of Bax has also been reported [32]. The E6 protein of HPV5 compromises the repair of UV-induced thymine dimers [33] and E6 of HPV7 forces keratinocytes into the S1-phase by inhibiting p53-activated, pro-apoptotic genes [34]. HPV8 E6 is able to bind XCRR1 that functions in a single strand DNA repair [35] and it has been shown that UV-irradiated cutaneous HPV8 E2-transgenic mice develop invasive carcinomatous lesions more rapidly than non-irradiated counterparts [36]. Moreover, E6/E7 expression of HPV20 influences proliferation and differentiation of the skin of UV-irradiated transgenic mice [37]. The anti-apoptotic activity and the delay of the DNA repair mechanism may lead to the persistence of UV-damaged keratinocytes, suggesting that cutaneous HPV types may be involved in the early stages of carcinogenesis.

A different mechanism behind the lack of cell cycle arrest in cutaneous HPV expressing cells is the up-regulation of ΔNp73 as a result of p53 accumulation observed in HPV38 E6 and E7 expressing human keratinocytes. ΔNp73 in turn inhibits the capacity of p53 to induce the transcription of genes involved in growth suppression [20], [21]. This observation, together with the efficiency of pRb binding and degradation by HPV38 E7, the HPV38 E6/E7-induced suboptimal activation of telomerase and the HPV38 E6/E7 transforming properties *in vivo* [38], seems to indicate that HPV38 E6 and E7, differently from proteins of other cutaneous HPV types, may be involved in the maintenance of oncogenic transformation.

The article "Interferon-β Induces Cellular Senescence in Cutaneous Human Papilloma Virus-Transformed Human Keratinocytes by Affecting p53 Transactivating Activity" was retracted in 2019. Reasons: manipulated images; duplicated images.

We have previously reported that type I IFNs inhibit cell proliferation in high risk mucosal HPV-positive Squamous Carcinoma Cell (SCC) lines by inducing a significant accumulation of cells in S-phase [24]. The S-phase deregulation triggers apoptotic cell death specifically mediated by the pro-apoptotic factor TRAIL [39].

The present study shows that IFN-β affects cell proliferation in keratinocytes expressing E6 and E7 proteins of cutaneous HPV-38 to a greater extent than in E6 and E7 mucosal HPV-16 transformed cells. In particular, K38 cells undergo senescence upon prolonged IFN-β treatment. IFN-β appears to induce senescence by up-regulating the expression of the tumor suppressor PML. Indeed, experiments of gene silencing via specific siRNAs have shown that PML is essential in the execution of senescence programme and that both p53 and p21 pathways are involved in senescence induction by IFN-β in K38 keratinocytes.

P53 and PML are critical mediators of senescence. PML is essential for the formation of discrete protein assemblages in the nucleus known as Nuclear Bodies (NBs) [40]. PML recruits into NBs p53 and proteins involved in p53 post-translational modifications that are essential for the activation of p53 and for the selection of target genes, such as the DNA damage responsive kinases ATM and ATR [25]. ATM kinase phosphorylates p53 at Ser-15, a senescence-inducible modification [41], in IFN-β-induced cellular senescence in human fibroblasts [16]. Over-expression of PML is capable of inducing premature senescence by stabilizing p53 via p53 acetylation on Lys-382 and phosphorylation on Ser-15 and Ser-46 [42]. In contrast, deacetylation of p53 antagonizes PML-induced premature senescence [43].

It has been shown that PML interacts with CBP/p300 acetyltransferase and stabilizes p53 through Lys-382 acetylation [42]. PML also recruits the tumor suppressor homeodomain-interacting protein kinase-2 (HIPK2) which induces p53Ser46 phosphorylation [44]. It has been reported that HIPK2-mediated phosphorylation of p53Ser46 is required for the CBP-induced p53 acetylation at Lys-382 [45]. PML has also been recently identified as a direct target of p53 revealing a regulatory positive feedback loop between p53 and PML [46].

The article "Interferon-β Induces Cellular Senescence in Cutaneous Human Papilloma Virus-Transformed Human Keratinocytes by Affecting p53 Transactivating Activity" was retracted in 2019. Reasons: manipulated images; duplicated images.

Our results indicate that in K38 cells p53 colocalyzes with IFN-β-induced PML into PML NBs. IFN-β can significantly modulate p53 phosphorylation at Ser-6,-15,-46, and -392 and acetylation status mainly at Lys-320. It has been also shown that p53 acetylation in Lys-320 is the first step in IFN-β-induced senescence in human fibroblasts [16].

DNA damage response is required for the activation of p53 in response to oncogenes. Oncogene induced senescence is accompained by DNA replicative stress, including prematurely terminated DNA replication forks and DNA double-strand breaks caused by hyper-DNA replication [47]. Consistent with this, Ras-induced senescence is associated with activation of DNA damage response effectors, such as ATM/ATR and Chk2/Chk1, and inactivation of these DNA damage effectors by RNA interference attenuates oncogene induced senescence [48], [49]. We observed that the inhibition of ATM and ATR prevents IFN-β induction of senescence in K38 keratinocytes, suggesting that IFN-β might induce senescence through a p53-dependent DNA damage pathway (data not shown).

It has been reported that HPV16 E6 mediates resistance to IFN-induced senescence through inhibition of p53 acetylation by binding to CBP/p300. Conversely, treatment of HPV16 E7-expressing cells with IFN ultimately resulted in cellular senescence through a process that is dependent upon acetylation of p53 by CBP/P300 [50]. Moreover, HPV16 E7 up-regulates SIRT1, thus attenuating p53 activity via its deacetylation [51]. It has been shown that HPV16 E6 can induce multiple site phosphorylation of p53 [52]. HPV38 E6 and E7 expression in human keratinocytes induces phosphorylation of p53, which leads to the up-regulation of ΔNp73 and the inhibition of p53 transcriptional induction of genes involved in growth suppression [21]. All together these observations indicate that p53 post-translational modifications are critical for p53 involvement in senescence programme induced by IFN-β and that modulation of p53 activity could be a common strategy utilized by both mucosal and cutaneous HPV to inhibit p53 function.

We report that by recruitment of p53 into NBs via PML induction, IFN-β may modulate p53 phosphorylation and acetylation status and downregulate ΔNp73 expression in K38 keratinocytes, leading to the recovery of p53 transactivating activity of selected target genes involved in cell proliferation control. Real time PCR array confirms that some genes involved in senescence and growth control are IFN-β-upregulated, in agreement with the reported observations [25] that modification of specific p53 phosphorylation and acetylation sites may correlate to the transactivation of growth related genes, suggesting a tissue and promoter-specific p53 activity regulation.

The article "Interferon-β Induces Cellular Senescence in Cutaneous Human Papilloma Virus-Transformed Human Keratinocytes by Affecting p53 Transactivating Activity" was retracted in 2019. Reasons: manipulated images; duplicated images.

Our results contribute to one of the most interesting current research questions about the exact contribution of post-translational modification sites to the selectivity of the global transcriptional programme of p53. Other important questions remain to be answered to clarify the multitude and redundancy of p53 covalent post-translational modifications required for p53-dependent senescence. It is possible that no single specific post-translational modification leads to specific p53 gene transactivation activity, but each modification might help to regulate p53 function in a tissue and promoter-specific manner.

## Materials and Methods

### Cell Cultures and Treatments

Primary human foreskin keratinocytes were transduced with empty retrovirus pLXSN (control), or with pLXSN38E6E7 or pLXSN16E6E7 as described by Caldeira et al., 2003 [20] and were grown in KBM BulletKit (Lonza).

HPV16-positive cell line Caski and SiHa, HPV18-positive cell line HeLa, and HPV68-positive cell line ME180, obtained from the American Type culture Collection, were grown in Dulbecco’s modified Eagle’s medium (DMEM) with 10% fetal bovine serum.

Cells were maintained in a humidified atmosphere of 5.5% CO_2_ at 37°C.

Human recombinant IFN-β (Rebif; 3×10^8^ IU/mg of protein; Ares-Serono) was added to the medium at the concentration of 200 IU/ml.

### Measurement of Cell Proliferation

Transformed keratinocytes were seeded in triplicate at 10^5^ cells per 35 mm dish. After 24 h, IFN-β was added to the cultures for the indicated times. Adherent cells were detached with 0.05% trypsin-0.02% EDTA in PBS, suspended in growth medium, and counted in a hemocytometer. Viability was evaluated by trypan blue exclusion.

### Flow Cytometry

For cell cycle analysis, cells were fixed in 70% ice-cold ethanol for at least 30 min. DNA staining was performed by incubating cells in PBS containing 0.18 mg/ml propidium iodide and 0.4 mg/ml DNase-free RNase. Cells were analysed on a FACScan flow cytometer (Becton and Dickinson).

### BrdU Incorporation

To determine the number of S-phase nuclei, cells were plated in triplicate at 10^5^ cells per 35 mm dish, treated with IFN-β for different time points and incubated with 50 µM BrdU for the last 5 hours. Samples were fixed with 95% ethanol, 5% acetic acid, treated with 1.5 M HCl and stained with an anti-BrdU monoclonal antibody (Amersham) followed by a rhodamine conjugated goat anti-mouse antibody (Cappel).

The article "Interferon-β Induces Cellular Senescence in Cutaneous Human Papilloma Virus-Transformed Human Keratinocytes by Affecting p53 Transactivating Activity" was retracted in 2019. Reasons: manipulated images; duplicated images.

### Senescence-associated β-galactosidase Staining

Cells were plated in 12 multi-well, 0,5×10^5^ cells per well, and treated with IFN-β at different time points. Senescent cells were quantified by counting cells displaying senescent-associated β-galactosidase activity at pH 6.0, assayed through Senescent Detection Kit (Calbiochem) following manufacturer’s instruction.

### Western Blot Analysis

To analyse protein expression, control and IFN-β treated cells were lysed in SDS reducing sample buffer. Total cell extracts were clarified by centrifugation and boiled in the presence of 5% 2-Mercaptoethanol and 0.01% bromophenol blue. Protein concentration was determined (Bio-Rad Protein Assay) and 30 mg of total proteins were resolved on SDS-PAGE and transferred onto PVDF membrane (Amersham). The membranes were blocked with 5% skim milk dissolved in PBS-T and incubated with primary antibodies (mouse anti-p53; rabbit anti-p21 (Santa Cruz); rabbit anti-PML (Bethyl); rabbit anti-phospho-p53 Ser6, anti-phospho-p53 Ser15, anti-phospho-p53 Ser46, anti-phospho-p53 Ser392 (Cell Signaling); rabbit anti-acetyl-p53 Lys320, anti-acetyl-p53 Lys373/382 (Millipore), and anti-human β tubulin mouse IgG1 antibody (ICN), as an internal control. Immune complexes were detected with horseradish peroxidase-conjugated goat anti-rabbit and anti-mouse antiserums (ICN) followed by enhanced chemiluminescence reaction (Millipore).

### PML, p53 and p21 silencing

Small interfering RNAs (siRNAs) targeted to PML, p53 and p21 were designed and validated by Qiagen and a non-silencing siRNA (Qiagen) served as control.

PML siRNAs were: 1) Sense:5′-CGUCUUUUUCGAGAGUCUGtt-3′;Antisense:5′-CAGACUCUCGAAAAAGACGtt-3′; 2)Sense:5′-CCCGCAAGACCAACAACAUtt-3′; Antisense: 5′-AUGUUGUUGGUCUUGCGGGtg-3′; 3)Sense:5′-GGGACCCUAUUGACGUUGAtt-3′; Antisense: 5′-UCAACGUCAAUAGGGUCCCtg-3′.

p53 siRNA were: 1) Sense:5′–GGAAAUUUGCGUGUGGAGUtt-3′; Antisense: 5′–CUCCACACGCAAAUUUCCtt-3′; 2) Sense: 5′-GCAUCUUAUCCGAGUGGAAtt-3′; Antisense: 5′-UUCCACUCGGAUAAGAUGCtg-3′; 3) Sense: 5′-GCAGUUAAGGGUUAGUUUAtt-3′; Antisense: 5′-UAAACUAACCCUUAACUGCaa-3′.

p21 siRNA (Dharmacon) was: Sense:5'-GAUGGAACUUCGACUUUGUUU-3': Antisense:5'-PACAAAGUCGAAGUUCCAUCUU 3'.

Shortly before transfection, 2×10^5^ cells per dish were seeded in 35 mm dishes in 1 ml of fully supplemented culture medium. siRNA was diluted in 50 µl culture medium without supplements to a final concentration of 10 nM. 3.5 µl of HiPerfect Transfection Reagent (Qiagen) were added to the diluted siRNA and mixed by vortexing. After an incubation of 10 min at room temperature, the transfection complex was added drop-wise onto the cells. 24 hrs post-transfection cells were treated with IFN-β for the indicated time points.

The article "Interferon-β Induces Cellular Senescence in Cutaneous Human Papilloma Virus-Transformed Human Keratinocytes by Affecting p53 Transactivating Activity" was retracted in 2019. Reasons: manipulated images; duplicated images.

### Immunofluorescence

Immunofluorescence staining of cells was performed on cells grown on Glass Bottom Culture Dishes 14 mm Microwell poly-d-lysine Coated from Mat Tek Corporation (Ashland, MA 01721 U.S.A.) and fixed with 4% formaldehyde, permeabilized with PBS/0.1% Triton-X, and stained using the following primary antibodies: anti-PML; ap53 (Santa Cruz), anti-ΔNp73 (Imgenex). Anti-mouse-Fitc (Cappel), anti-mouse-Alexa 546 (Molecular Probe # A11030), and anti-rabbit-Alexa 610 (Molecular Probe # A31551) were used as secondary antibodies. Sample were analyzed using confocal microscope (Leica TCS SP5). Software: LAS AF version 1.6.3 (Leica Microsystem).

### Real-time PCR

Real-time PCR was carried out by using the MESA GREEN MasterMixes Plus, Low ROX (Eurogentec). The primer sequences are: Bax F: 5' TTT GCT TCA GGG TTT CAT CC 3', R: 5' ATC CTC TGC AGC TCC ATG TT 3'; Pig3 F: 5' GCT TCA AAT GGC AGA AAA GC 3', R: 5' AAC CCA TCG ACC ATC AAG AG 3'.
